# Xiaoxuming Decoction Regulates Vascular Function by Modulating G Protein-Coupled Receptors: A Molecular Docking Study

**DOI:** 10.1155/2021/5575443

**Published:** 2021-06-05

**Authors:** Yanjia Shen, Ran Yang, Rui Zhou, Wendan Lu, Li Li, Ziran Niu, Miao Chen, Jinhua Wang, Yuehua Wang, Lianhua Fang, Guanhua Du

**Affiliations:** ^1^Beijing Key Laboratory of Drug Targets Identification and Drug Screening, Institute of Materia Medica, Chinese Academy of Medical Sciences and Peking Union Medical College, Beijing, China; ^2^Biomedical Engineering Research Center, Kunming Medical University, Kunming, China; ^3^Department of Pharmacy, Peking Union Medical College Hospital, Chinese Academy of Medical Sciences and Peking Union Medical College, Beijing, China

## Abstract

Xiaoxuming decoction (XXMD) is a traditional Chinese herbal medicine (CHM) that is used for the treatment of stroke in China. Stroke injury damages the cerebral vasculature and disrupts the autoregulation of vasoconstriction and vasodilatation, which is crucial for maintaining constant cerebral blood flow (CBF). It has been reported that XXMD exerts a positive effect on cerebral circulation in animal models of stroke. However, the mechanisms underlying the regulatory effect of XXMD on vascular tone, and the interactions among the multiple components of XXMD, remain unclear. In this study, XXMD was found to induce relaxation of the basilar artery rings of rats precontracted by 5-hydroxytryptamine (5-HT) *in vitro*, in a dose-dependent manner. The modulation of vascular tone and the process of cerebral ischemia are mediated via the interactions between G protein-coupled receptors (GPCRs) and their ligands, including 5-HT, angiotensin II (Ang II), and urotensin II (UII). Thus, the potential synergistic effects of the different components of XXMD on the regulation of vasoconstriction and vasodilation were further investigated by molecular docking based on network pharmacology. We constructed and analyzed a database comprising 963 compounds of XXMD and studied the interactions between five vascular GPCRs (5-HT1A receptor (5-HT1AR), 5-HT1B receptor (5-HT1BR), Ang II type 1 receptor (AT1R), beta 2-adrenergic receptor (*β*2-AR), and UII receptor (UTR)) and the various herbal constituents of XXMD using molecular docking. By constructing and analyzing the compound-target networks of XXMD, we found that *Glycyrrhizae Radix et Rhizoma*, *Ginseng Radix et Rhizoma*, and *Paeoniae Radix Alba* were the three major herbs that contained a large number of compounds with high docking scores. We additionally observed that several constituents of XXMD, including gallotannin, liquiritin apioside, nariutin, 1,2,3,4,6-pentagalloylglucose, folic acid, and ginsenoside Rb1, targeted multiple vascular GPCRs. Moreover, the interactions between the components of XXMD and the targets related to vascular tone constituted the comprehensive cerebrovascular regulatory function of XXMD and provided a material basis of the vasoregulatory function of XXMD. The study reports the contributions of various components of XXMD to the regulatory effects on vascular tone and provides scientific evidence for the multicomponent and multitargeting characteristics of XXMD.

## 1. Introduction

Xiaoxuming decoction (XXMD) is a well-known traditional Chinese herbal medicine (CHM), which was recorded in Beiji Qianjin Yaofang, written by Sun Simiao of the Tang Dynasty, and has been widely used for over centuries in China to treat strokes in clinics [1]. This formula consists of twelve Chinese herbs, including *Scutellariae Radix*, *Paeoniae Radix Alba*, *Glycyrrhizae Radix et Rhizoma*, *Stephaniae Tetrandrae Radix*, *Ginseng Radix et Rhizoma*, *Cinnamomi Ramulus*, *Armeniacae Semen Amarum*, *Ephedrae Herba*, *Chuanxiong Rhizoma*, *Aconiti Lateralis Radix Praeparata*, *Saposhnikoviae Radix*, and *Zingiberis Rhizoma Recens* at a 1 : 1 : 1 : 1 : 1 : 1 : 1 : 1 : 1 : 1 : 1.5 : 5 ratio. Preclinical studies from our laboratory and other groups have demonstrated that XXMD has neuroprotective effects in rats with acute or chronic cerebral ischemia [2–10]. The anti-ischemic activity of XXMD is mediated via numerous mechanisms, including the inhibition of oxidative stress [2], reduction of neuronal apoptosis [3], preservation of mitochondrial integrity and improvement of mitochondrial function [4, 5], reduction in the activity of inducible nitric oxide synthase (iNOS) in cerebral tissues [6], alleviation of blood-brain barrier (BBB) disruption [7], protection of the neurovascular unit [8], suppression of astrocyte activation [9], and regulation of the expression of differentially expressed proteins in the hippocampus [10]. Notably, a meta-analysis of eight randomized controlled trials (RCTs) published between 1992 and 2012 revealed that XXMD improves neurological deficits and is safe in patients with acute ischemic stroke when compared to Western conventional medicine (WCM), which was used as the control [1]. However, the mechanisms underlying the activity of XXMD in the treatment of stroke remain unclear.

Stroke is a type of acute cerebral vascular disease, which is the leading cause of adult disability and the second most common cause of death worldwide [11]. Stroke occurs when the blood supply to a part of the brain is interrupted, and the brain cells die due to oxygen or nutrient insufficiency. There are two main categories of stroke, namely, ischemic stroke, in which the flow of blood is restricted, and hemorrhagic stroke, which is characterized by bleeding. Ischemia induces cerebral damage, which impairs the vasculature and adversely affects cerebral blood flow (CBF) [12]. As insufficient blood supply is presently considered to be a major pathology of stroke, drugs that induce recovery of the cerebral blood supply are of enormous promise. The drugs that modulate the vascular tone and dilate the cerebral arteries can restore blood supply to the ischemic area and thus provide a material basis for the subsequent antireperfusion injury and neuronal protection.

G protein-coupled receptors (GPCRs), also known as seven-transmembrane domain receptors, can regulate vascular contraction by activating second messengers, including cyclic adenosine monophosphate (cAMP), inositol trisphosphate (IP_3_), and Ca^2+^ [13]. It is known that 5-hydroxytryptamine (5-HT), angiotensin II (Ang II), and urotensin II (UII) are strong vasoconstrictors and regulate blood pressure. These substances can trigger vasoconstriction by binding to their specific receptors, including 5-HT 1A receptor (5-HT1AR), 5-HT1B receptor (5-HT1BR), Ang II type 1 receptor (AT1R), and UII receptor (UTR) [14–16]. Beta 2-adrenergic receptor (*β*2-AR) can alter the tension of blood vessels and regulate the release of renin [17, 18]. Accumulating evidence has demonstrated that both GPCRs and their ligands, including 5-HT, Ang II, and UII, partake in the process of cerebral ischemia [19–21]. XXMD exerts a positive effect on cerebral vasculature and circulation in animal models of stroke [9, 22, 23]. Previous studies have demonstrated that XXMD increases regional CBF in experimental rats with cerebral hemorrhage [24] and also improves the reduction in cerebrovascular reactivity induced by chronic cerebral ischemia in rats [9]. However, the underlying mechanisms and interactions between the constituents of XXMD and vascular GPCRs are yet to be fully understood.

Network pharmacology is based on the theory of systems biology and is used to perform network analysis of biological systems. In network pharmacology, a specific signal node (nodes) can be selected to perform novel analyses of a multitarget drug for molecular design. Network pharmacology can serve as a robust method for studying “drugs-target-disease” networks, which may be closer to elucidating the complex nature of the disease being investigated [25]. To date, network-based methods have been used as a novel strategy for discovering the constituents of traditional Chinese medicine (TCM), identifying bioactive compounds, and elucidating the mechanisms underlying the action of herbal formulae [26]. Molecular docking is a computer-assisted approach that is primarily used to study the interactions between two or several molecules using both geometric complementarity and energy matches. Molecular docking has been widely used in drug discovery and serves as an important tool for the investigation and evaluation of herbal medicines [27, 28]. The combined use of molecular docking and network pharmacology can provide valuable information and improve the accuracy of the prediction.

Although some progress has been made in the pharmacological investigation of XXMD over the past few years [1–10, 29], the interactions among the multiple components of XXMD remain to be elucidated. The investigation of TCM using network pharmacology can aid in the discovery of multiple therapeutic targets for the various active ingredients to formulate effective interactions and therapeutic targets. This approach can be used to identify the targets, the group of active constituents that play a role in the interactions, and the material basis of the active herbal components of XXMD.

In this study, we found that XXMD could induce relaxation of the basilar artery rings of rats precontracted by 5-HT in a dose-dependent manner. However, the mechanism underlying the modulation of vascular tone and the material basis of XXMD remain unclear. We performed molecular docking for investigating the potential synergistic effects of the constituents of different herbs in XXMD on the regulation of vascular tone. The interactions between the five GPCRs linked to vasoconstriction (5-HT1AR, 5-HT1BR, AT1R, *β*2-AR, and UTR) and the various herbal constituents of XXMD were assessed. The compound-target networks for XXMD were subsequently constructed and analyzed.

## 2. Materials and Methods

### 2.1. Preparation of XXMD

All the twelve crude herbs of XXMD were purchased from Beijing Tongrentang Co., Ltd. (Beijing, China). The identification and deposition of these medicinal herbs and the preparation of XXMD were performed by Jiangsu Kanion Pharmaceutical Co., Ltd. (China). Briefly, the crude herbs were soaked in 95% aqueous ethanol for 2 hours and refluxed in a heated water bath for 1 hour. The filtered and mixed suspensions were collected, and their concentrations were subsequently determined. The extraction was performed thrice using petroleum ether. The fraction eluted with 40% ethanol and the intermediate layer fraction were incorporated into XXMD [10].

### 2.2. Preparation of Rat Cerebral Arterial Rings

Male Sprague–Dawley rats, weighing 240-260 g, were provided by Vital River Laboratories (Beijing, China). The animals were housed in plastic cages under controlled humidity and temperature and were exposed to a 12-hour light/dark cycle. The animals had *ad libitum* access to purified water and a standard diet. Animal care and handling were performed in accordance with the guidelines of the Institutional Animal Care and Use Committee of the Chinese Academy of Medical Science and Peking Union Medical College.

The rats were euthanized by cervical dislocation, following which the basilar artery was rapidly isolated and cut into 2 mm long segments in ice-cold physiological saline solution (PSS) having the following composition (mmol/L): NaCl 130, KCl 4.7, MgSO_4_ 1.17, KH_2_PO_4_ 1.18, NaHCO_3_ 14.9, glucose 5.5, ethylene diamine tetraacetic acid 0.026, and CaCl_2_ 1.6. For intact tissue preparation, extreme care was taken to avoid endothelial cell damage. The segments were then mounted on 40 *μ*m stainless steel wires in a Multi Myograph System (Danish Myograph Technology, Aarhus, Denmark), and the contractile responses were determined. The organ chamber was filled with 5 mL of PSS, through which 95% O_2_/5% CO_2_ was continually bubbled, and the temperature was maintained at 37°C. The segments of the basilar arteries were normalized to the optimal initial tension, according to the instructions provided with the Multi Myograph System. The segments were then allowed to equilibrate for 60 min at the resting tension. The PSS was changed every 20 min during equilibration. After equilibration, the arterial rings were constricted twice with a high K^+^ (60 mmol/L) PSS (K-PSS) having the following composition (mmol/L): NaCl 74.7, KCl 60, MgSO_4_ 1.17, KH_2_PO_4_ 1.18, NaHCO_3_ 14.9, glucose 5.5, ethylene diamine tetraacetic acid 0.026, and CaCl_2_ 1.6. The integrity of a functional endothelium was verified by the ability of acetylcholine (Ach) (20 *μ*mol/L) to induce more than 60% relaxation in the arterial rings precontracted with 60 mmol/L K-PSS [30].

### 2.3. 5-HT-Induced Contraction in Isolated Cerebral Arterial Rings

The basilar arterial rings with intact endothelium were precontracted with 1 *μ*mol/L 5-HT (Sigma). After a sustained contraction was obtained, XXMD was added to the bathing solution in a cumulative manner (1, 3, 10, 30, 100, 200, 300, and 400 *μ*g/mL) to obtain the concentration-response curves.

### 2.4. Retrieval of the Constituents of XXMD

The chemical constituents of the twelve herbs in XXMD were retrieved from China Natural Product Database (http://pharmdata.ncmi.cn) and from the literature. The chemical structures were drawn using ISIS Draw 2.5 (MDL Information Systems, Inc.).

### 2.5. Preparation of Ligands and Target Proteins

Five vascular GPCRs (5-HT1AR, 5-HT1BR, AT1R, *β*2-AR, and UTR) were considered for the molecular docking study. The crystal structures of 5-HT1BR, AT1R, and *β*2-AR were retrieved from the RCSB Protein Data Bank (PDB) (http://www.pdb.org/) [31], and the PDB codes were 4IAQ, 4YAY, and 4LDE, respectively. The structures of the GPCRs for which crystal structures were unavailable, namely, 5-HT1AR and UTR, were constructed by homology modeling using Discovery Studio 4.1. After sequence comparison, the sequences of *β*2-AR (PDB ID: 2RH1) and 5-HT1BR (PDB ID: 4IAQ) were selected as the templates for modeling UTR and 5-HT1AR, respectively. The Build Homology Model module in Discovery Studio was used for homology modeling, and the model with optimal reliability was selected for molecular docking.

A ligand library, comprising the different conformations of each ligand, was constructed using the Prepare Ligands tool. The existing ligands and water of crystallization in the target proteins were removed using the Prepare Protein tool. The ligand-receptor binding sites were determined using the Define and Edit Binding Site tool, based on the information obtained from the binding sites of the cocrystallized ligands in the protein structures. For 5-HT1BR and AT1R, the binding sites of the cocrystallized ligands, dihydroergotamine and 5,7-diethyl-1-{[2′-(1H-tetrazol-5-yl) biphenyl-4-yl]methyl}-3,4-dihydro-1,6-naphthyridin-2(1H)-one, respectively, were defined as the active ligand-binding pocket. For *β*2-AR, the binding site of BI167107 was defined as the active ligand-binding pocket.

### 2.6. Molecular Docking

The LibDock module of Dock Ligands in Discovery Studio 4.1 was used to perform molecular docking. The conformation method was set to fast to ensure docking accuracy and velocity, and the other parameters were set to default. In this semiflexible docking approach, 100 or less conformations of each ligand were generated to ensure computational speed and comprehensiveness. The output index and LibDock scores were subsequently obtained. The scores indicate the binding affinity between the receptors and the ligand conformations. The higher the score of a small molecule, the stronger the protein binding affinity. For each target, the 50 top-scoring compounds were selected, and their scores were considered to be the highest among all the conformations for each ligand. The LibDock scores of the agonists and antagonists, retrieved from the IUPHAR database, were also determined for each target, for assessing the potential activity of the herbal compounds in XXMD. The following agonists and antagonists were used for molecular docking: 5-HT1AR (agonists: U92016A, vilazodone, and vortioxetine; antagonists: (S)-UH 301 and WAY-100635); 5-HT1BR (agonists: CP94253, eletriptan, and L-694,247; antagonists: GR-55562 and SB236057); AT1R (agonists: L-162,313; antagonists: candesartan, irbesartan, and valsartan), *β*2-AR (agonists: formoterol, salmeterol, and zinterol; antagonists: carvedilol, propranolol, and timolol; and UTR (agonists: AC-7954 and FL104; antagonists: palosuran and SB-706375).

### 2.7. Compound-Target Network Construction Using Cytoscape

The information pertaining to the chemical composition and related compound-target network interactions were analyzed using Cytoscape version 3.7.1. The compound-target network was established using Cytoscape, and the interactions were subsequently visualized.

## 3. Results

### 3.1. XXMD Induces Relaxation of Rat Basilar Artery Rings Precontracted by 5-HT

XXMD was found to induce relaxation of the rat basilar artery rings (Figure 1). The maximum relaxant effect of XXMD on the rings precontracted by 5-HT was 97.13 ± 2.74%. The pEC50 value was 4.44 ± 0.09.

### 3.2. Construction and Analysis of the Compound Database of XXMD

In order to identify the potential material basis of the modulatory effects of XXMD on the vascular tone, 963 compounds from the twelve herbs of XXMD were retrieved from China Natural Product Database and from the literature. The number of compounds in each herb was determined, and the results are depicted in Figure 2. The compounds were subsequently classified on the basis of their chemical structures, and the distribution of the compounds among the different chemical categories is provided in Table 1 and Figure 3. The results demonstrated that the five top-ranking chemical categories in the prescription were essential oils (32%), flavonoids (24%), alkaloids (13%), saponins (7%), phenols, and organic acids (5%). However, it should be noted that the results reflect the number of different types of compounds rather than their abundance or relative content in the prescription.

In order to identify the potentially effective constituents of XXMD, the compounds derived from the different herbs of XXMD were retrieved and analyzed. The names, plant sources, and chemical categories of forty compounds are enlisted in Table 2. Of the compounds that were derived from multiple plant sources, the majority were essential oils, flavonoids, phenols, or organic acids. This result was consistent with the data pertaining to the major chemical constituents of XXMD.

### 3.3. Molecular Docking of Ligands to Vascular GPCR Targets

The cocrystallized ligands were redocked to the five vascular GPCR targets (5-HT1AR, 5-HT1BR, AT1R, *β*2-AR, and UTR) using the LibDock program in Discovery Studio 4.1. The ligands dihydroergotamine, 5,7-diethyl-1-{[2′-(1H-tetrazol-5-yl) biphenyl-4-yl]methyl}-3,4-dihydro-1,6-naphthyridin-2(1H)-one, and BI167107 were extracted from the crystal structures of 5-HT1BR, AT1R, and *β*2-AR, respectively, and redocked into the active site of the corresponding receptors. The root mean square deviation (RMSD) values between the docked poses and the ligand conformation in the crystallographic complexes were 0.3074, 0.3168, and 0.4324 Å, which indicated that the docking protocol was highly accurate and reliable.

For each GPCR target, the compounds with the highest scores were selected to generate a scatter diagram, as depicted in Figure 4. The LibDock scores of the agonists and antagonists of the GPCR targets are provided in Figure 4. Most of the chemical constituents of XXMD could be successfully docked to the target GPCRs. For each GPCR, some of the compounds exhibited higher LibDock scores than the agonists and antagonists, indicating their strong binding affinity to the GPCR targets. Nevertheless, some of the compounds failed to dock to the target GPCRs owing to their structural characteristics.

In order to analyze the overall results of ligand-receptor docking, we determined the number of compounds that were successfully docked and the percentage of compounds with LibDock scores higher than the average scores of the agonists and antagonists. As demonstrated in Table 3, 76.52%, 84.46%, 84.89%, 76.96%, and 78.70% of the compounds in XXMD successfully docked to 5-HT1AR, 5-HT1BR, AT1R, *β*2-AR, and UTR, respectively. Additionally, more than 10% of the compounds of XXMD had higher LibDock scores than the average score of the GPCR agonists and antagonists. Therefore, these results suggested that most of the compounds of XXMD have the potential to bind and interact with the five vascular GPCRs considered herein. It subsequently follows that the vascular tone can be comprehensively modulated by XXMD via the interactions between the multiple chemical constituents of XXMD and the different vascular GPCR targets in the compound-target network.

### 3.4. Construction and Analysis of Compound-Target Interaction Network of XXMD

In order to elucidate the material basis of the modulation of vascular tone by XXMD, the 50 top-scoring compounds that targeted the vascular GPCRs were selected, and the compound-target network of XXMD was constructed using Cytoscape version 3.7.1. As depicted in Figure 5, the blue and yellow nodes represent the chemical components and targets, respectively, while the edges represent the interactions. The network analyzer plugin of Cytoscape was used to analyze the network by calculating the number of nodes, network density, and network heterogeneity, among other factors. The compound-target network comprised 249 edges, 135 nodes, 130 compounds (after removal of duplicates), and 5 targets. Network analysis revealed that multiple compounds targeted the same GPCR, while some of the compounds had multiple targets, which demonstrated that the perspective of CHM is very different from the philosophy of WCM, which considers that one compound interacts with one specific target.

In order to explore the relationships between the chemical constituents of the twelve herbs of XXMD and the five vascular GPCR targets, the 50 top-scoring compounds with the highest docking scores were selected for each of the targets and categorized according to their herbal sources (Figure 6). The three major herbs were *Glycyrrhizae Radix et Rhizoma*, *Ginseng Radix et Rhizoma*, and *Paeoniae Radix Alba*.

The compound-target network interactions were subsequently analyzed. Several of the 50 top-scoring compounds interacted with multiple targets, including 5-HT1AR, 5-HT1BR, AT1R, *β*2-AR, and UTR. As depicted in Figure 7 and Table 4, 3 compounds of XXMD, namely, gallotannin, liquiritin apioside, and narirutin, interacted with all the five GPCRs, while 11 compounds, including 1,2,3,4,6-pentagalloylglucose and folic acid, interacted with 4 targets. On the other hand, 19 compounds, including ginsenoside Rb1, interacted with 3 GPCR targets, and 36 compounds interacted with 2 of the GPCR targets. The binding modes of gallotannin, liquiritin apioside, and nariutin in the binding sites of the GPCR targets (5-HT1AR, 5-HT1BR, AT1R, *β*2-AR, and UTR) are depicted in Figure 8, Figure 9, and Figure 10, respectively.

## 4. Discussion

To date, there are no definitive treatment strategies for ischemic stroke. With the development of recent research on multi-component-multi-target drugs, the functions of TCM in the treatment of complex diseases have become increasingly important. Owing to the potent compound group formulation used in TCM prescriptions, the efficacy of TCM is attributed to the interactions between multiple active ingredients and multiple disease targets. Several animal experiments and clinical studies have demonstrated that XXMD, a CHM with relaxant effects on cerebral blood vessels, can improve the treatment outcomes in both acute and chronic ischemic brain injury [4, 5, 10]. By relaxing the cerebral blood vessels, XXMD can restore the supply of blood and nutrients to the ischemic area, providing a material basis of the prevention of reperfusion injury and neuronal protection.

In this study, the vasorelaxant effects of XXMD on rat basilar arteries contracted by 5-HT were determined. The modulation of vascular tone and the process of cerebral ischemia are mediated via the interactions between GPCRs and their ligands, including 5-HT, Ang II, and UII. Therefore, molecular docking was performed to determine the potential synergistic effects of the components of XXMD on the regulation of vascular tone via modulation of the activity of vascular GPCRs. First, a database of 963 compounds of XXMD, with different chemical structures, was constructed and analyzed. Molecular docking was used to investigate the interactions between the chemical constituents of XXMD and the five vascular GPCRs, namely, 5-HT1AR, 5-HT1BR, AT1R, *β*2-AR, and UTR. The 50 top-scoring compounds with high docking scores to each of the GPCR targets were selected and sorted. The herbal sources of these compounds were determined for identifying the roles of the twelve herbs of XXMD in regulating the vascular tone via modulation of GPCR activity.

The results of our study suggested that several overlapping compounds and their analogues are widely distributed in the different medicinal herbs of XXMD. The contents of these ingredients are relatively high in the XXMD prescription, compared to those of the other compounds. Furthermore, previous studies have demonstrated that most of these compounds have similar physiological activities, including antitumor, anti-inflammatory, antioxidative, neuroprotective, blood lipid-regulating, and vasorelaxant properties. These compounds, derived from a variety of different plants in XXMD, have different chemical structures and can produce synergistic therapeutic effects under the same pathological conditions. Therefore, they are likely to be the key components that play a crucial role in the therapeutic effect of XXMD.

Apart from their pharmacological activities, some of the chemical ingredients, including essential oils, promote the absorption of other drugs. It is speculated that ginger is indispensable in the treatment of cerebral apoplexy by XXMD, and the maximum dosage should be five *Liang* [32]. Furthermore, it has been demonstrated that ginger extract improves memory deficits and neuronal density in rats with focal cerebral ischemia [33]. It can therefore be concluded that the essential oils, which are the main chemical components of ginger, are likely to enhance the absorption of other constituents in several CHMs.

Classification of the herbal sources of the 50 top-scoring compounds revealed that the three major herbs were *Glycyrrhizae Radix et Rhizoma*, *Ginseng Radix et Rhizoma*, and *Paeoniae Radix Alba*. The therapeutic potential of these herbs and their constituents in cerebral ischemia has been extensively studied. It has been demonstrated that the aqueous extract of licorice (*Glycyrrhizae Radix et Rhizoma*) reduces infarct volumes and exerts a neuroprotective effect by regulating the expression of apoptosis-related proteins in mice with middle cerebral artery occlusion (MCAO) [34]. Glycyrrhizin (GL) [35] and 18*β*-glycyrrhetinic acid (GA) [36], isolated from the roots of licorice, have also been reported to have neuroprotective effects in focal cerebral ischemia/reperfusion brain injury, which are mediated via the anti-inflammatory, antioxidant, and antiapoptotic effects of GL, or the strong antioxidant and radical scavenging properties of GA in global cerebral ischemia/reperfusion brain injury. Isoliquiritigenin (ISL), a flavonoid present in the roots of licorice, is known to have vasorelaxant effects and protects against injury due to cerebral ischemia by ameliorating cerebral energy metabolism and via its antioxidant properties [37]. Ginsenoside Rd, belonging to the class of *Ginseng Radix et Rhizoma* compounds in herbal medicine, has been shown to attenuate damage due to ischemic stroke via suppression of oxidative stress and inflammation [38]. The active metabolite of ginsenosides in the gut, 20(S)-protopanaxadiol, induces vasorelaxation in isolated rat thoracic aorta via an endothelium-independent pathway [39]. A combination of *Paeoniae Radix Alba* and *Rhizoma Ligustici Chuanxiong* was reported to ameliorate focal cerebral ischemia in rats with MCAO by attenuating the endoplasmic reticulum stress-dependent apoptotic signaling pathway [40]. Therefore, the results of this study indicate that *Glycyrrhizae Radix et Rhizoma*, *Ginseng Radix et Rhizoma*, and *Paeoniae Radix Alba* play a key role in the modulatory effect of XXMD on vascular tone and its effects on suppressing ischemic stroke via regulation of the compound-target interaction network in XXMD and necessitate further investigation.

It has been reported that TCM influences disease progression by modulating GPCR activity. The Chinese herbal formula, Sini Tang (SNT), comprises *Glycyrrhizae Radix et Rhizoma*, *Aconiti Lateralis Radix Praeparata*, and *Zingiberis Rhizoma Recens*. SNT improves cardiac function by inhibiting the excessive activation of the renin-angiotensin-aldosterone system, which involves a reduction in the levels of plasma angiotensin II and downregulation of the protein and gene levels of AT1R in heart failure after myocardial infarction in rats [41]. ISL has also been reported to exhibit *in vitro* 5-HT2B receptor antagonistic activity [42]. Ginsenoside Rb1 has been reported to possess antidepressant-like activity, which is mediated via the modulation of 5-HT_2A_ receptors [43]. The results of our study demonstrated that XXMD inhibited the constriction of rat basil artery induced by 5-HT. However, the effects of XXMD on vasoconstriction induced by other GPCR ligands, and the underlying mechanism involving the modulation of GPCRs and their signaling pathways, necessitate further investigation.

By reviewing the relevant literature, we found that most of the components of XXMD that target multiple vascular GPCRs possess vasorelaxant effects and suppress ischemic stroke. For instance, 1,2,3,4,6-pentagalloylglucose, a major component of *Paeoniae Radix Alba*, binds to 4 vascular GPCR targets and has been reported to induce vasorelaxation and suppress the vascular inflammatory process by activating the NO/cGMP signaling pathway [44]. Folic acid, a member of the vitamin B complex, and isolated from *Ginseng Radix et Rhizoma* and *Chuanxiong Rhizoma*, was found to bind to 4 GPCR targets. Interestingly, folic acid has been reported to improve endothelial function [45] and alleviate various microglia-mediated neuroinflammation via the Notch1/nuclear factor kappa B p65 pathway in the hippocampus following brain I/R injury in rats [46]. Ginsenoside Rb1, an active component extracted from *Ginseng Radix et Rhizoma*, was found to bind to three GPCR targets and has been reported to promote poststroke axonal regeneration by activating the cAMP/PKA/CREB signaling pathway [47]. Few studies have investigated the vasorelaxant and anti-ischemic stroke effects of the three compounds of XXMD, namely, gallotannin, liquiritin apioside, and narirutin, which bound to all the five vascular GPCR targets. It is therefore necessary to study the effects of these three compounds in further detail. The results of our study demonstrate that the compounds that targeted the vascular GPCRs could mediate the modulatory effect of XXMD on vascular tone and provide a material basis of the treatment of ischemic stroke with XXMD. However, the results of this study need to be verified using experiments and data validation.

In conclusion, the current study clearly demonstrated that XXMD was able to relax the cerebral artery rings of rats. XXMD comprises numerous compounds with different chemical structures and is derived from multiple plant sources. Therefore, XXMD might regulate cerebrovascular function via the network of interactions between the constituents of XXMD and the GPCRs involved in vasoconstriction. Our results demonstrated that the various herbal constituents of XXMD contribute to the regulation of vascular tone via the modulation of the target GPCRs. By investigating and analyzing the monomeric component of XXMD from the perspective of chemical composition and the relationships between the chemical constituents and targets, we were able to provide evidence for understanding the mechanisms underlying the effect of XXMD in the treatment of stroke.

## Figures and Tables

**Figure 1:** Vasorelaxant effects of XXMD on endothelium-intact basilar artery precontracted with 5-HT. The results are presented as the mean ± standard error of mean (SEM); *n* = 7.

**Figure 2:** Number of compounds in the herbal constituents of XXMD.

**Figure 3:** Classification and proportion of the chemical constituents of XXMD.

**Figure 4:** LibDock scores obtained by molecular docking of the chemical constituents of XXMD with the five vascular GPCR targets. The five vascular GPCR targets are (a) 5-HT1AR, (b) 5-HT1BR, (c) AT1R, (d) *β*2-AR, and (e) UTR.

**Figure 5:** Compound-target interaction network of XXMD. The blue and yellow nodes represent the chemical constituents and targets, respectively, while the edges represent the interactions. The network was constructed and visualized using Cytoscape 3.7.1.

**Figure 6:** Enrichment of the 50 top-scoring compounds with high docking scores with each of the vascular GPCR targets, classified according to their herbal source in XXMD.

**Figure 7:** The number of top 50 scoring compounds that interacted with multiple vascular GPCR targets.

**Figure 8:** The binding modes of gallotannin in the ligand-binding site of (a) 5-HT1AR, (b) 5-HT1BR, (c) AT1R, (d) *β*2-AR, and (e) UTR.

**Figure 9:** The binding modes of liquiritin apioside in the ligand-binding site of (a) 5-HT1AR, (b) 5-HT1BR, (c) AT1R, (d) *β*2-AR, and (e) UTR.

**Figure 10:** The binding modes of nariutin in the ligand-binding site of (a) 5-HT1AR, (b) 5-HT1BR, (c) AT1R, (d) *β*2-AR, and (e) UTR.

**Table 1:** Classification and number of chemical constituents in XXMD.

Classification	Number	Classification	Number
Essential oils	309	Coumarin	23
Flavonoids	232	Tannins	16
Alkaloid	124	Chromone	15
Saponin	69	Polyacetylene	14
Phenol and organic acid	49	Steroid	12
Fatty acid and ester	28	Others	44
Glycosides	28	In total	963

**Table 2:** The overlapping chemicals that are derived from different herbs in XXMD.

Compound	Plant source	Chemical classification	Compound	Plant source	Chemical classification
1,8-Cineole	*Ephedrae Herba, Zingiberis Rhizoma Recens*	A	Bornylene	*Cinnamomi Ramulus, Saposhnikoviae Radix*	A
2-Nonanone	*Saposhnikoviae Radix, Zingiberis Rhizoma Recens*	A	Camphene	*Saposhnikoviae Radix root, Zingiberis Rhizoma Recens*	A
2-Nonenal	*Armeniacae Semen Amarum, Saposhnikoviae Radix,*	A	Camphor	*Armeniacae Semen Amarum, Zingiberis Rhizoma Recens*	A
3-Carene	*Chuanxiong Rhizoma, Zingiberis Rhizoma Recens*	A	Caryophyllene	*Armeniacae Semen Amarum, Ginseng Radix et Rhizoma, Zingiberis Rhizoma Recens*	A
Alloaeromadendrene	*Ginseng Radix et Rhizoma, Zingiberis Rhizoma Recens*	A	Citral	*Armeniacae Semen Amarum, Zingiberis Rhizoma Recens*	A
Alpha-cadinene	*Chuanxiong Rhizoma, Zingiberis Rhizoma Recens*	A	Gamma-elemene	*Ginseng Radix et Rhizoma, Zingiberis Rhizoma Recens*	A
Benzaldehyde	*Armeniacae Semen Amarum, Cinnamomi Ramulus*	A	Hexanal	*Armeniacae Semen Amarum, Saposhnikoviae Radix*	A
Beta-bisabolene	*Ginseng Radix et Rhizoma, Saposhnikoviae Radix, Zingiberis Rhizoma Recens*	A	Limonene	*Chuanxiong Rhizoma, Ephedrae Herba*	A
Beta-elemene	*Armeniacae Semen Ginseng Radix et Rhizoma, Zingiberis Rhizoma Recens*	A	Naphthaline	*Ephedrae Herba, Saposhnikoviae Radix*	A
Beta-eudesmol	*Saposhnikoviae Radix, Zingiberis Rhizoma Recens*	A	Nonanaldehyde	*Armeniacae Semen Amarum, Saposhnikoviae Radix root*	A
Borneol	*Armeniacae Semen Amarum, Cinnamomi Ramulus, Zingiberis Rhizoma Recens*	A	Terpineol	*Ephedrae Herba, Zingiberis Rhizoma Recens*	A
Eriodictyol	*Armeniacae Semen Amarum, Scutellariae Radix*	B	Caffeic acid	*Chuanxiong Rhizoma, Ephedrae Herba*	E
Kaempferol	*Cinnamomi Ramulus, Glycyrrhizae Radix et Rhizoma, Paeoniae Radix Alba*	B	Cinnamic acid	*Cinnamomi Ramulus, Ephedrae Herba*	E
Quercetin	*Ephedrae Herba, Glycyrrhizae Radix et Rhizoma*	B	Folic acid	*Chuanxiong Rhizoma, Ginseng Radix et Rhizoma*	E
Rutin	*Ephedrae Herba, Glycyrrhizae Radix et Rhizoma*	B	Malic acid	*Ephedrae Herba, Ginseng Radix et Rhizoma*	E
Wogonin	*Saposhnikoviae Radix, Scutellariae Radix*	B	Protocatechuic acid	*Cinnamomi Ramulus, Chuanxiong Rhizoma, Ephedrae Herba*	E
Choline	*Chuanxiong Rhizoma, Ginseng Radix et Rhizoma*	C	Daucosterol	*Aconiti Lateralis Radix Praeparata, Ginseng Radix et Rhizoma, Paeoniae Radix Alba, Saposhnikoviae Radix*	F
Chuanxiongzine	*Chuanxiong Rhizoma, Ephedrae Herba*	C	Panaxynol	*Ginseng Radix et Rhizoma, Saposhnikoviae Radix*	G
Linoleic acid	*Ephedrae Herba, Stephaniae Tetrandrae Radix*	D	Beta-sitosterol	*Aconiti Lateralis Radix Praeparata, Cinnamomi Ramulus, Paeoniae Radix Alba, Saposhnikoviae Radix*	H
Palmitic acid	*Chuanxiong Rhizoma, Ephedrae Herba, Saposhnikoviae Radix, Stephaniae Tetrandrae Radix*	D	Campesterol	*Ginseng Radix et Rhizoma, Scutellariae Radix*	H

A: essential oil; B: flavonoid; C: alkaloid; D: saponin; E: phenol and organic acid; F: fatty acid and ester; G: polyacetylene; H: Steroid.

**Table 3:** Overview of the LibDock scores of the chemical constituents of XXMD with the five vascular GPCRs.

%	5-HT1AR	5-HT1BR	AT1R	*β*2-AR	UTR
Docked ratio	76.52	84.46	84.89	76.96	78.70
> positive mean ratio	34.78	13.37	10.54	11.74	10.65

**Table 4:** The compounds in XXMD that interacted with multiple targets.

No.	Compounds	Source	The number of targets
1	Gallotannins	*Paeoniae Radix Alba*	5
2	Liquiritin apioside	*Glycyrrhizae Radix et Rhizoma*	5
3	Narirutin	*Glycyrrhizae Radix et Rhizoma*	5
4	1,2,3,4,6-Pentagalloylglucose	*Paeoniae Radix Alba*	4
5	20(R)-Ginsenoside Rg2	*Ginseng Radix et Rhizoma*	4
6	Chrysin-6-C-*α*-L-arabinopyranosyl-8-C-*β*-D-glucopyranoside	*Scutellariae Radix*	4
7	Eugeniin	*Paeoniae Radix Alba*	4
8	Folic acid	*Ginseng Radix et Rhizoma, Chuanxiong Rhizoma*	4
9	Gingerglycolipid B	*Cinnamomi Ramulus*	4
10	Gingerglycolipid C	*Cinnamomi Ramulus*	4
11	Licoagrone	*Glycyrrhizae Radix et Rhizoma*	4
12	Inflasaponin IV	*Glycyrrhizae Radix et Rhizoma*	4
13	Paeonidanin C	*Paeoniae Radix Alba*	4
14	Paeonidanin E	*Paeoniae Radix Alba*	4
15	(2S)-1-O-(9Z,12Z-Octadeeadienoly)-3-O-*β*-D-galactopyranosyl-glycerol	*Cinnamomi Ramulus*	3
16	1,2,3,6-Tetra-O-gafloyl-*β*-D-glucose	*Paeoniae Radix Alba*	3
17	1-O-Galloylpedunculagin	*Paeoniae Radix Alba*	3
18	2-(3-Hydroxy-4-methoxyphenyl)-ethyl-1-O-*α*-L-rhamnosyl-(1 ⟶ 3)-*β*-D-(4-feruloyl)-glucoside	*Scutellariae Radix*	3
19	3-O-*β*-D-Glucopyranosyl betulinic acid-28-O-*β*-D-glucopyranosyl-(1 ⟶ 6)-*β*-D-glucopyranoside	*Ginseng Radix et Rhizoma*	3
20	5,7,4^″^-Trihydroxy-6-C-arabinoside-8-C-glucoside flavone	*Scutellariae Radix*	3
21	6,5′-dipernylluteolin	*Glycyrrhizae Radix et Rhizoma*	3
22	Argininyl-fructosyl-glucose	*Ginseng Radix et Rhizoma*	3
23	Delsemine B	*Aconiti Lateralis Radix Praeparata*	3
24	Demethyldelavaine B	*Aconiti Lateralis Radix Praeparata*	3
25	Ginsenoside Rb1	*Ginseng Radix et Rhizoma*	3
26	Isoliquiritin apioside	*Glycyrrhizae Radix et Rhizoma*	3
27	Licoagroside F	*Glycyrrhizae Radix et Rhizoma*	3
28	Licoricesaponine F3	*Glycyrrhizae Radix et Rhizoma*	3
29	Liquiritigenin-7,4^″^-diglucoside	*Glycyrrhizae Radix et Rhizoma*	3
30	Mahuangnin B	*Ephedrae Herba*	3
31	Methyl-n-buthy-uralsaponin A esters	*Glycyrrhizae Radix et Rhizoma*	3
32	n-Triacontanol	*Ephedrae Herba*	3
33	Vicenin-2	*Glycyrrhizae Radix et Rhizoma, Ephedrae Herba*	3
34	(Z)-(1S,5R)-*β*-Pinen-l0-yl-*β*-vicianoside	*Paeoniae Radix Alba*	2
35	3-Hydroxyglabrol II	*Glycyrrhizae Radix et Rhizoma*	2
36	5-Epicatechin	*Cinnamomi Ramulus*	2
37	6′-Malonylginsenoside Rd1	*Ginseng Radix et Rhizoma*	2
38	Amygdalin	*Armeniacae semen Amarum*	2
39	Araloside A	*Ginseng Radix et Rhizoma*	2
40	Daucosterol	*Ginseng Radix et Rhizoma, Paeoniae Radix Alba, Saposhnikoviae Radix, Aconiti Lateralis Radix Praeparata*	2
41	Delsemine A	*Aconiti Lateralis Radix Praeparata*	2
42	Demethyldelavaine A	*Aconiti Lateralis Radix Praeparata*	2
43	Dibutyl uralsaponin A esters	*Glycyrrhizae Radix et Rhizoma*	2
44	Dihydrobaicalin	*Scutellariae Radix*	2
45	Gancaonin E	*Glycyrrhizae Radix et Rhizoma*	2
46	Gingerenone B	*Zingiberis Rhizoma Recens*	2
47	Ginsenoside La	*Ginseng Radix et Rhizoma*	2
48	Ginsenoside Rb3	*Ginseng Radix et Rhizoma*	2
49	Ginsenoside Rg3	*Paeoniae Radix Alba*	2
50	Glycyroside	*Glycyrrhizae Radix et Rhizoma*	2
51	Gnetin H	*Paeoniae Radix Alba*	2
52	Isotrilobine	*Stephaniae Tetrandrae Radix*	2
53	Isotrilobine-N-2-oxide	*Stephaniae Tetrandrae Radix*	2
54	Licoagrodin	*Glycyrrhizae Radix et Rhizoma*	2
55	Licoricesaponine A3	*Glycyrrhizae Radix et Rhizoma*	2
56	Licoricesaponine C2	*Glycyrrhizae Radix et Rhizoma*	2
57	Licoricesaponine D3	*Glycyrrhizae Radix et Rhizoma*	2
58	Licoricesaponine H2	*Glycyrrhizae Radix et Rhizoma*	2
59	Licoricesaponine K2	*Glycyrrhizae Radix et Rhizoma*	2
60	Liquiritigenin-7-O-*β*-D-(3-O-acetyl)-apiofuranosyl-4^″^-O-*β*-D-glucopyranoside	*Glycyrrhizae Radix et Rhizoma*	2
61	Mahuangnin D	*Ephedrae Herba*	2
62	Meso-3,5-diacetoxy-1,7-bis-(4-hydroxy-3-methoxyphenyl)heptanes	*Zingiberis Rhizoma Recens*	2
63	Nonacosanol	*Ephedrae Herba*	2
64	Paeonidanin A	*Paeoniae Radix Alba*	2
65	Paeonidanin B	*Paeoniae Radix Alba*	2
66	Paeonidanin D	*Paeoniae Radix Alba*	2
67	Scutellarin	*Scutellariae Radix*	2
68	Uralsaponin A	*Glycyrrhizae Radix et Rhizoma*	2
69	Vlcenin-2	*Glycyrrhizae Radix et Rhizoma*	2

## Data Availability

The data used to support the findings of this study are included within the article. Other data are available from the corresponding author upon request.
